The article "Effect of LAMA4 on Prognosis and Its Correlation with Immune Infiltration in Gastric Cancer" was published in 2021. Journal: Biomed Res Int.

# Effect of LAMA4 on Prognosis and Its Correlation with Immune Infiltration in Gastric Cancer

**DOI:** 10.1155/2021/6428873

**Published:** 2021-08-09

**Authors:** Mingming Wang, Changzheng Li, Ying Liu, Zuomin Wang

**Affiliations:** ^1^Department of Medical Oncology, Shandong Cancer Hospital and Institute, Shandong First Medical University and Shandong Academy of Medical Sciences, Jiyan Road 440, Jinan, 250117 Shandong, China; ^2^Department of Oncology, Central Hospital Affiliated to Shandong First Medical University, Jiefang Road 105, Jinan, 250013 Shandong, China

## Abstract

**Background:**

Laminin alpha 4 (LAMA4) is widely distributed in the basement membranes of various tissues. It can regulate cancer cell proliferation and migration. We investigated the effects of LAMA4 in gastric cancer (GC).

**Methods:**

LAMA4 expression patterns were analyzed in GC using the Gene Expression Omnibus (GEO), Gene Expression Profiling Interactive Analysis (GEPIA), and UALCAN. Correlations between LAMA4 expression and clinicopathological characteristics were evaluated using data from The Cancer Genome Atlas (TCGA). The survival analysis was examined using the Kaplan-Meier plotter and GEPIA and ascertained by multivariate Cox analysis. Genetic alterations and DNA methylation of LAMA4 were analyzed using cBioPortal and MethSurv. LinkedOmics was applied to identify coexpressed genes of LAMA4. The association between LAMA4 and infiltration of immune cells was explored using Tumor Immune Estimation Resource (TIMER) and GEPIA.

**Results:**

LAMA4 was highly expressed in GC, and its upregulation significantly correlated with T classification (*P* = 0.040). LAMA4 expression was an independent risk factor for overall survival (OS, *P* = 0.033). Patients with genetic alterations of LAMA4 showed a significantly better disease-free survival (DFS, *P* = 0.022). Ten CpG sites of LAMA4 were significantly associated with prognosis in GC. The functions of LAMA4 and coexpression genes were mainly involved in extracellular matrix (ECM) receptor interaction. LAMA4 expression significantly correlated with infiltration of macrophages (*P* < 0.001), CD4+ T cells (*P* < 0.001), and dendritic cells (*P* < 0.001). Furthermore, LAMA4 expression was significantly associated with markers of M2 and tumor-associated macrophages (TAMs).

**Conclusion:**

LAMA4 expression was linked to GC prognosis and immune cell infiltration, indicating its potential use as a prognostic biomarker and therapeutic target.

## 1. Introduction

Gastric cancer (GC) is one of the most aggressive and deadliest types of cancers. The relatively late detection and high recurrence potential of GC contribute to its high mortality rate. The development of targeted therapy and immunotherapy facilitated individualized treatment and improved prognosis for GC patients [1]. However, existing treatment results remain disappointing due to the heterogeneity of tumors. Little is known about the carcinogenic and host factors that drive tumor progression or induce drug resistance. Therefore, identification of effective diagnostic and prognostic factors could be instrumental in improving current therapy strategies for GC patients, thus extending survival.

The article "Effect of LAMA4 on Prognosis and Its Correlation with Immune Infiltration in Gastric Cancer" was published in 2021. Journal: Biomed Res Int.

Laminin alpha 4 (LAMA4), a component of the laminin family, is mainly distributed in endothelial and some epithelial basement membranes [2]. It plays a significant role in mediating cell adhesion and migration, as well as organizing cells into tissues during embryonic development by interacting with other extracellular matrix (ECM) components [3]. Over recent decades, the effects of LAMA4 on cancers have attracted wide attention. LAMA4 was shown to be specifically upregulated in hepatocellular carcinoma and was significantly correlated with tumor invasion and metastasis [4]. LAMA4 expression was found to be increased in breast cancer cells and associated with cancer initiation and progression [5]. High expression levels of LAMA4 were also shown to predict poor survival in renal cell carcinoma [6]. On the contrary, LAMA4 was markedly downregulated in ovarian cancer, and overexpression of LAMA4 significantly impaired ovarian cancer cell proliferation, invasion, and migration [7]. In GC, LAMA4 was reported to be associated with enhanced cisplatin resistance and poor overall survival (OS) [8, 9]. However, the mechanisms and functions of LAMA4 are not fully understood in GC.

The present study analyzed the expression levels of LAMA4 in GC using data available in public databases. The associations between LAMA4 expression and clinicopathologic features and OS were evaluated. The molecular changes of LAMA4, including genetic alterations and DNA methylation, and their impacts on survival were explored. Coexpression genes that may be involved in GC progression were screened using LinkedOmics analysis. Finally, the relationship between LAMA4 expression and tumor immune infiltration was investigated. Our results provide evidence for the role of LAMA4 in GC carcinogenesis and prognosis and may help to identify a potential biomarker for GC prognosis and therapy.

## 2. Materials and Methods

### 2.1. Data Acquisition

The four gene expression profiles GSE13911, GSE54129, GSE79973, and GSE19826 were obtained from the Gene Expression Omnibus (GEO). GSE13911 contained 38 GC tumor samples and 31 normal gastric samples. GSE54129 contained 111 GC tumor samples and 21 normal gastric samples. GSE79973 contained 10 paired GC and adjacent normal gastric samples. GSE19826 contained 12 paired GC and adjacent normal gastric samples. The raw data were normalized using the affy package in R language [10]. The clinicopathological and survival data of GC from The Cancer Genome Atlas (TCGA) were downloaded using the UCSC Xena browser [11].

The article "Effect of LAMA4 on Prognosis and Its Correlation with Immune Infiltration in Gastric Cancer" was published in 2021. Journal: Biomed Res Int.

### 2.2. Expression and Survival Analysis

The expression differences from two groups included in each of the four profiles from GEO were displayed in plots through GraphPad Prism 8. The expression levels of LAMA4 between GC and normal gastric tissues in TCGA were analyzed in the Gene Expression Profiling Interactive Analysis (GEPIA) and UALCAN databases [12, 13]. The Kaplan-Meier plotter and GEPIA database were used to compare the survival differences between high and low LAMA4 expression groups in GC.

### 2.3. Genetic Alterations and DNA Methylation Analysis

The cBioPortal database was applied to analyze the genetic alterations of LAMA4 in GC [14]. A MethSurv web tool was applied to analyze the DNA methylation data of LAMA4 and evaluate the prognostic value of each CpG site in GC [15].

### 2.4. Coexpression Genes of LAMA4

The genes coexpressed with LAMA4 in GC were screened using the LinkFinder module of the LinkedOmics database [16]. The results were displayed in the form of volcano and heat plots. Through Gene Set Enrichment Analysis (GSEA) of the LinkInterpreter module, Gene Ontology (biological process) and Kyoto Encyclopedia of Genes and Genomes (KEGG) pathways were identified. GEPIA was applied to plot survival heatmaps of the top 50 coexpression genes.

### 2.5. Immune Infiltrate Correlation Analysis

Associations between LAMA4 expression and six infiltrating immune cells (B cells, CD4+ T cells, CD8+ T cells, neutrophils, macrophages, and dendritic cells) were explored using the Tumor Immune Estimation Resource (TIMER) platform [17]. The purity-corrected partial Spearman's correlation (partial-cor) and *P* value were displayed in scatter plots. Multivariate Cox analysis was used to evaluate the effect of LAMA4 and immune cells on survival. Moreover, the associations between LAMA4 expression and gene markers of tumor-associated macrophages (TAMs) and M1 and M2 macrophages were analyzed in TIMER and GEPIA. The gene markers were obtained from related references [18–22].

### 2.6. Statistics

SPSS 25.0 was used for statistical analyses. An independent sample *t*-test and a paired sample *t*-test were used to compare the differential expression levels of LAMA4 between the GC tissues and nontumor tissues. The Pearson chi-squared test was used to assess the association between LAMA4 expression and clinicopathological variables. Univariate and multivariate Cox proportional hazards regression models were used to calculate the hazard ratio (HR), 95% confidence interval (CI), and the correlation between LAMA4 expression level and OS. *P* < 0.05 was considered statistically significant.

The article "Effect of LAMA4 on Prognosis and Its Correlation with Immune Infiltration in Gastric Cancer" was published in 2021. Journal: Biomed Res Int.

## 3. Results

### 3.1. LAMA4 Expression Levels in GC

LAMA4 expression levels were assessed in GC tissues and normal gastric tissues from four GEO dataset profiles. Unpaired and paired groups consistently showed that LAMA4 mRNA expression levels were significantly upregulated in tumor samples compared with nontumor tissues (all *P* < 0.05, Figures 1(a) – 1(d)). This tendency was also found in TCGA cohorts using GEPIA and UALCAN databases, although the differences were not statistically significant (Figures 1(e) and 1(f)).

### 3.2. Correlations between LAMA4 Expression and Clinicopathological Characteristics

Correlations between LAMA4 expression and clinical variables of GC in TCGA were evaluated using 319 GC samples with LAMA4 expression and clinical information. A total of 160 samples were classified as high, and 159 were low based on the median values of LAMA4 expression levels. These results indicated that LAMA4 expression was significantly different among different cancer grades (*P* = 0.031, Table 1). Moreover, high levels of LAMA4 expression were observed as T classification increased (*P* = 0.040, Table 1). However, no significant association was found between LAMA4 expression and age, gender, stage, and N and M classification.

### 3.3. LAMA4 Is an Independent Predictor of Worse OS in GC

Differences in OS were compared between the high and low LAMA4 expression groups in GC using the Kaplan-Meier plotter with GEO data and the GEPIA platform with TCGA data to assess the value of LAMA4 as a prognostic biomarker. The high LAMA4 expression group showed a significantly shorter OS than the low expression group in both GEO data (*P* < 0.001, Figure 2(a)) and TCGA data (*P* = 0.003, Figure 2(b)). Univariate Cox analysis of TCGA data indicated that age, gender, TNM stage, N classification, and LAMA4 expression were significant risk factors for survival (all *P* < 0.05, Table 2). Multivariate Cox analysis confirmed the critical role of age (*P* = 0.003) and LAMA4 expression (*P* = 0.033) as independent predictors of unfavorable OS for GC (Figure 2(c)). Therefore, LAMA4 may be a potential independent prognostic factor in GC.

### 3.4. Genetic Alterations and DNA Methylation of LAMA4

Genetic alterations and DNA methylation were analyzed to gain a deeper understanding of the molecular mechanism of LAMA4. Genetic alterations were seen in 8% of the 393 samples, with mutation, deletion, and amplification as the most common events (Figure 3(a)). Patients with genetic alterations of LAMA4 showed a significantly better disease-free survival (DFS) than those without alterations (*P* = 0.022, Figure 3(b)). However, there was no difference in OS between the two groups (Figure 3(c)). The DNA methylation heatmap of LAMA4 is shown in Figure 4(a). Among the 20 CpG sites, cg16044777 showed the highest levels of methylation. The prognostic value of each CpG site was evaluated. High levels of DNA methylation in 10 CpGs were significantly associated with better OS in GC (Table 3). As shown in Figures 4(b) – 4(k), the survival difference between the higher and lower DNA methylation levels of cg11934419 was the most pronounced (*P* = 4.9*e* − 05).

The article "Effect of LAMA4 on Prognosis and Its Correlation with Immune Infiltration in Gastric Cancer" was published in 2021. Journal: Biomed Res Int.

### 3.5. Coexpression Networks of LAMA4

LinkedOmics was used to investigate the coexpression profiles with LAMA4 in GC. A total of 7765 genes and 5711 genes were positively and negatively correlated with LAMA4, respectively (Figure 5(a)). The top 50 genes that were positively and negatively coexpressed with LAMA4 in GC are shown in Figures 5(b) and 5(c), respectively. Gene Ontology analysis carried out by GSEA revealed that the genes coexpressed with LAMA4 were mainly involved in the following biological process: extracellular structure organization, cyclic nucleotide metabolic process, and vasculogenesis (Figure 5(d)). KEGG pathway analysis showed that the genes were primarily enriched in ECM-receptor interaction, hypertrophic cardiomyopathy, and Hedgehog signaling pathway (Figure 5(e)). Notably, 25 of the top 50 positively correlated genes and 8 of the top 50 negatively correlated genes showed remarkable high and low hazard ratios, respectively, for GC survival (Figures 5(f) and 5(g)).

### 3.6. Association of LAMA4 Expression with Immune Cell Infiltration

We further analyzed whether LAMA4 expression was correlated with the infiltration of six major types of immune cells. Our results showed that LAMA4 expression was significantly positively correlated with infiltration of macrophages (*r* = 0.636, *P* = 2.07*e* − 43), CD4+ T cells (*r* = 0.448, *P* = 1.70*e* − 19), and dendritic cells (*r* = 0.422, *P* = 2.03*e* − 17) in GC (Figure 6(a)). The multivariate Cox hazards model was used to assess the impact of LAMA4 expression and the six types of immune cells on the OS of GC. Overall, macrophages (*P* = 0.003) were significantly related to OS (Table 4).

### 3.7. Correlation Analysis between LAMA4 Expression and Macrophage Immune Marker Genes

Since LAMA4 expression showed a strong positive association with macrophage infiltration, we focused on the correlation between LAMA4 expression and marker genes of different macrophage subtypes. After adjustment for tumor purity, we found a significant correlation between LAMA4 expression and markers of M2 macrophages and TAMs. Expression of CD163, MS4A4A, and MRC1 of M2 macrophages and CCL2, CD68, and IL10 of TAMs showed a significantly positive correlation with LAMA4 expression (all *P* < 0.001, Figures 6(b) and 6(c)). M1 macrophage markers, such as PTGS2, NOS2, and ARG2, showed a weak or no correlation with LAMA4 expression (Figure 6(d)). In addition, we assessed the relationship between these markers and LAMA4 expression in the GEPIA database and consistently found the same positive trend in M2 macrophages and TAMs (Table 5).

The article "Effect of LAMA4 on Prognosis and Its Correlation with Immune Infiltration in Gastric Cancer" was published in 2021. Journal: Biomed Res Int.

## 4. Discussion

Despite great advances in the treatment strategies of GC, long-term survival remains poor. Delayed diagnosis, frequent drug resistance, and rapid recurrence account for the limited benefits of treatment. The molecular characteristics of GC remain to be fully elucidated. Probing valuable prognostic and therapeutic targets is urgently required to optimize individualized treatment and improve prognosis. The present study analyzed differences in LAMA4 expression between GC and normal gastric groups in multiple datasets. LAMA4 was upregulated in GC tissues, and high levels of LAMA4 expression were significantly correlated with tumor invasion. Univariate and multivariate Cox analysis indicated that age and LAMA4 upexpression were independent predictors of unfavorable OS in GC.

LAMA4, known as a basement membrane glycoprotein, promotes the migration, proliferation, and survival of endothelial, blood, and cancer cells [23–25]. LAMA4 mRNA and protein expression was shown to be elevated in triple-negative breast cancer [26]. Pancreatic cancer patients with higher levels of LAMA4 expression were more likely to have liver metastasis and worse survival [27]. Knockdown of LAMA4 suppressed glioma cell adhesion and migration and reduced cell invasiveness [28]. It has been suggested that miR-539 and miRNA-200b could negatively regulate LAMA4 expression by directly targeting its 3′-untranslated regions [26, 29]. In the present study, evaluation of the differential expression in GC revealed that LAMA4 was highly expressed in tumor samples. Higher expression levels of LAMA4 were found more frequently with higher T classification. Survival analysis in GEO and TCGA samples indicated that high LAMA4 expression was associated with worse OS. Further multivariate Cox analysis confirmed LAMA4 as an independent risk factor for prognosis in GC. Hence, LAMA4 may be a valuable diagnostic and prognostic biomarker that should be studied further in detail.

The article "Effect of LAMA4 on Prognosis and Its Correlation with Immune Infiltration in Gastric Cancer" was published in 2021. Journal: Biomed Res Int.

We next explored the possible genetic and epigenetic alterations of LAMA4 in GC. According to the cBioPortal, genetic alterations of LAMA4 were found in 8% of the GC samples. The mutation was the most frequent phenomenon. DNA methylation analysis indicated that CpGs with higher methylation levels were mainly focused in Open_Sea and N_Shelf of LAMA4, whereas CpGs with lower methylation levels were common in Island and S_Shore. Interestingly, patients with genetic alterations exhibited a better DFS than those without. CpG sites located in the LAMA4 Island were all significantly associated with prognosis. Taken together with the survival advantage in the low expression group, we propose that genetic or epigenetic alterations may induce LAMA4 disorders as GC progresses. It was reported that low methylation of LAMA4 was associated with a significantly poor progression-free survival in ovarian cancer [30]. LAMA4 DNA methylation levels were negatively correlated with the tumor histologic grade in pancreatic cancer patients [27]. Further studies are needed to elucidate the mechanisms underlying genetic and epigenetic modifications of LAMA4 and their associations with expression in GC.

Coexpression analysis was performed to determine the biological functions of LAMA4. Our results revealed that LAMA4 and related coexpression genes were primarily enriched in extracellular structure organization and ECM-receptor interaction pathway. As a member of ECM glycoproteins, LAMA4 is ubiquitously localized in endothelial basement membranes. Disruption of LAMA4 expression inhibited endothelial sprouting and tubulogenesis [31]. It was reported that LAMA4 could impact the behavior of endothelial cells via complex interactions with integrin receptors on the surface of endothelial cells [32]. LAMA4 secreted from pancreatic cancer cells was shown to have a positive influence on the migration of fibroblasts in the tumor microenvironment [27]. LAMA4 overexpression induced cell migration in renal cell carcinoma via activation of the ILK/FAK/ERK pathway [29]. In GC cells, LAMA4 knockdown led to a reduced tumor invasive capability via inhibiting the expression of MMP2, a critical enzyme that degrades ECM [9]. Taken together, these findings indicate that LAMA4 plays an important role in regulating GC tumorigenesis via cell-matrix interactions.

Cumulative evidence indicates that immune cell infiltration can affect the progression and prognosis of GC [33, 34]. We evaluated the correlation between LAMA4 expression and immune cell infiltration in GC. LAMA4 expression was strongly and favorably associated with infiltration of macrophages. Cox analyses showed that macrophage was a significantly independent risk factor among all variables. In addition, LAMA4 expression also correlated with most molecular markers of macrophage subtypes in GC. The analysis based on the TIMER database showed that gene markers of the M2 macrophage strongly correlated with LAMA4 expression, whereas TAM markers exhibited moderate and M1 macrophage markers exhibited weak correlations. The correlations above were checked in the GEPIA database. Together, the results suggested a potential function of LAMA4 in TAM polarization. TAM infiltration in GC is closely related to tumorigenesis and metastasis and affects the survival rate of GC patients [35–37]. TAM may polarize into M1 or M2 macrophages in response to microenvironmental signals [38]. M2 macrophages play an important role in promoting metastasis via epithelial mesenchymal transition promotion in GC cells and facilitating gastric tumor proliferation and progression [39, 40]. The results above suggested the hypothesis that high expression of LAMA4 may accelerate GC progression and affect prognosis via regulation of TAMs.

The article "Effect of LAMA4 on Prognosis and Its Correlation with Immune Infiltration in Gastric Cancer" was published in 2021. Journal: Biomed Res Int.

At present, how LAMA4 affects the prognosis of GC and the function of LAMA4 in GC has not been fully elaborated. Our study provided new insights into the possible role of LAMA4 in GC. However, there are some limitations. All the data analyzed were retrospective and from multiple public datasets, which were not verified by our own experiments. More effort is needed to explore the detailed mechanisms of LAMA4 in GC.

## 5. Conclusions

In conclusion, we identified that increased LAMA4 expression in GC predicted adverse prognosis. Genetic and methylation alterations of LAMA4 affected DFS and OS in GC, respectively. LAMA4 expression was closely associated with infiltration of immune cells, particularly macrophages. LAMA4 might be a potential prognostic biomarker and therapeutic target in GC.

## Figures and Tables

**Figure 1:** The expression levels of LAMA4 in gastric cancer (GC). (a–d) LAMA4 expression comparisons between GC and nontumor tissues from 4 GEO profiles. (e, f) LAMA4 expression comparisons between GC and nontumor tissues from TCGA samples evaluated by GEPIA (*P* > 0.05) (e) and UALCAN (*P* > 0.05) (f). GEO: Gene Expression Omnibus; TCGA: The Cancer Genome Atlas.

**Figure 2:** High expression of LAMA4 is associated with worse survival in GC. (a) Survival analysis of LAMA4 in the GEO dataset using the Kaplan-Meier plotter. (b) Survival analysis of LAMA4 in the TCGA samples using GEPIA. (c) Multivariate Cox analysis of the correlation between LAMA4 expression and survival. HR: hazard ratio; CI: confidence interval.

**Figure 3:** Genetic alterations of LAMA4 and the association between alterations and survival. (a) Genetic alterations of LAMA4 in GC using cBioPortal. (b) GC patients with LAMA4 genetic alterations showed a better DFS than those without (*P* = 0.0222). (c) Genetic alterations of LAMA4 did not have an impact on OS in GC (*P* = 0.351). DFS: disease-free survival; OS: overall survival.

The article "Effect of LAMA4 on Prognosis and Its Correlation with Immune Infiltration in Gastric Cancer" was published in 2021. Journal: Biomed Res Int.

**Figure 4:** The heatmap of LAMA4 DNA methylation and the prognostic value of DNA methylation. (a) The heatmap of CpG methylation levels of LAMA4. Red to blue: high levels of DNA methylation to low levels. (b–k) High methylation level of cg16044777 (b), cg23082393 (c), cg00491418 (d), cg16267162 (e), cg09105802 (f), cg01254555 (g), cg04555779 (h), cg13938098 (i), cg08897388 (j), and cg11934419 (k) correlated with better OS.

**Figure 5:** Coexpression genes of LAMA4 in GC. (a) Volcano plot of genes highly correlated with LAMA4 identified by the Spearman test in GC. Red and green dots represent genes significantly positively and negatively correlated with LAMA4, respectively. (b, c) Heatmaps of the top 50 genes positively (b) and negatively (c) correlated with LAMA4. (d, e) Significantly enriched GO: biological process annotations and KEGG pathways of LAMA4. (f, g) Survival heatmaps of the top 50 genes positively (f) and negatively (g) correlated with LAMA4 using GEPIA. The survival heatmaps are presented in the form of a logarithmic scale (log10) of hazard ratios. The red and blue squares indicate higher and lower risks for survival, respectively. The bordered squares indicate the significant unfavorable and favorable survival (*P* < 0.05). GO: Gene Ontology; KEGG: Kyoto Encyclopedia of Genes and Genomes.

**Figure 6:** Correlations between LAMA4 expression and six infiltrating immune cells and subtypes of macrophage in GC. (a) LAMA4 expression was significantly positively correlated with infiltration of CD4+ T cells, macrophages, and dendritic cells. (b) Correlations of LAMA4 expression with marker genes of the M2 macrophage (CD163, MS4A4A, and MRC1). (c) Correlations of LAMA4 expression with marker genes of TAM (CCL2, CD68, and IL10). (d) Correlations of LAMA4 expression with marker genes of the M1 macrophage (PTGS2, NOS2, and ARG2). TAM: tumor-associated macrophage; TPM: transcript per million.

**Table 1:** Relationship between LAMA4 expression level and clinicopathological variables in gastric cancer.

Classification	Total	LAMA4 expression		*χ* ^2^	*P* value
		High	Low		
Age					
60	218	111	107	0.159	0.690
<60	101	49	52		
Gender					
Female	120	56	64	0.937	0.333
Male	199	104	95		
Grade					
G1	7	4	3	6.936	0.031
G2	110	44	66		
G3	202	112	90		
TNM stage					
I	44	17	27	2.710	0.100
II-IV	275	143	132		
T classification					
T1	16	4	12	8.319	0.040
T2	64	28	36		
T3	152	76	76		
T4	87	52	35		
N classification					
N0	101	48	53	2.075	0.557
N1	83	39	44		
N2	69	35	34		
N3	66	38	28		
M classification					
M0	297	149	148	0.000	0.988
M1	22	11	11		

The article "Effect of LAMA4 on Prognosis and Its Correlation with Immune Infiltration in Gastric Cancer" was published in 2021. Journal: Biomed Res Int.

**Table 2:** Univariate analysis of the prognostic factors in gastric cancer patients using a Cox regression model.

Variables	Univariate analysis		
	HR	95% CI	*P* value
Age, year (≥60, <60)	1.665	1.114-2.489	0.013
Gender (male vs. female)	1.469	1.001-2.154	0.049
Grade (G3 vs. G1-G2)	1.282	0.887-1.854	0.186
TNM stage (III-IV vs. I-II)	1.718	1.189-2.481	0.004
T classification (T3-T4 vs. T1-T2)	1.455	0.936-2.263	0.096
N classification (N1-N3 vs. N0)	1.704	1.114-2.608	0.014
M classification (M1 vs. M0)	1.626	0.851-3.108	0.141
LAMA4 expression (high vs. low)	1.624	1.138-2.316	0.008

**Table 3:** The prognostic values of CpG sites in LAMA4.

CpG	Relation to CpG island	RefGene group	HR	*P* value
cg00491418	Island	5′UTR	0.582	0.0011
cg04555779	Island	5′UTR	0.596	0.0017
cg16267162	Island	5′UTR	0.615	0.0033
cg01254555	Island	Body	0.641	0.029
cg09105802	Island	Body	0.651	0.035
cg25567805	N_Shelf	Body	0.699	0.072
cg16044777	Open_Sea	Body	0.627	0.0051
cg23082393	Open_Sea	Body	0.595	0.01
cg12188410	Open_Sea	Body	0.737	0.094
cg16689724	Open_Sea	3′UTR	0.771	0.11
cg08191490	Open_Sea	Body	0.763	0.16
cg09414426	Open_Sea	Body	1.241	0.19
cg04204246	Open_Sea	Body	0.8	0.25
cg03106852	Open_Sea	Body	1.149	0.47
cg05512869	Open_Sea	Body	1.091	0.59
cg11934419	S_Shore	TSS200	0.495	0.000049
cg08897388	S_Shore	1st exon; 5′UTR	0.56	0.0045
cg13938098	S_Shore	TSS200	0.686	0.022
cg14289461	S_Shore	TSS200	0.748	0.076
cg08844365	S_Shore	TSS1500	0.835	0.35

**Table 4:** The multivariate Cox proportional hazards model of LAMA4 and six tumor-infiltrating immune cells in GC (TIMER).

	Coefficient	HR	95% CI	*P* value
Purity	-0.485	0.616	0.303-1.251	0.180
B cell	3.404	30.094	0.373-2427.743	0.129
CD8+ T cell	-1.387	0.250	0.015-4.067	0.330
CD4+ T cell	-4.270	0.014	0.000-1.464	0.072
Macrophage	5.201	181.393	5.932-5546.629	0.003
Neutrophil	1.175	3.237	0.008-1324.515	0.702
Dendritic	0.254	1.289	0.083-19.967	0.856
LAMA4	0.138	1.148	0.930-1.416	0.198

**Table 5:** Correlation analysis between LAMA4 expression and maker genes of macrophage subtypes (GEPIA).

	Marker	*R*	*P* value
M2 macrophage	CD163	0.48	1.30*E* − 24
	MS4A4A	0.53	5.50*E* − 31
	MRC1	0.54	1.10*E* − 32

TAM	CCL2	0.54	9.60*E* − 32
	CD68	0.31	2.50*E* − 10
	IL10	0.49	3.60*E* − 26

M1 macrophage	PTGS2	0.4	1.90*E* − 17
	NOS2	0.067	0.18
	ARG2	-0.064	0.2

## Data Availability

All the data used in the current study are available from the public database, and they can be found in the Gene Expression Omnibus (https://www.ncbi.nlm.nih.gov/geo/), The Cancer Genome Atlas (https://xenabrowser.net/datapages/), the cBioPortal (https://www.cbioportal.org/), the MethSurv (https://biit.cs.ut.ee/methsurv/), the LinkedOmics (http://www.linkedomics.org/), and the Tumor Immune Estimation Resource (https://cistrome.shinyapps.io/timer/).
